The article "Analysis of Nursing Effect of Children with Henoch-Schonlein Purpura Based on the PDCA Nursing Model" was retracted in 2022. Reason: concerns about the peer review.

# Analysis of Nursing Effect of Children with Henoch-Schonlein Purpura Based on the PDCA Nursing Model

**DOI:** 10.1155/2021/1736429

**Published:** 2021-12-13

**Authors:** Shuai Qin, Dan Li, Bo Zhang

**Affiliations:** Tangshan Workers Hospital, Tangshan 063000, China

## Abstract

By applying the PDCA model to the care of children with Henoch-Schonlein purpura, the nursing process can be divided into four stages: planning, execution, inspection, and treatment. According to the age characteristics and disease progression of pediatric patients, a complete nursing plan is formulated to efficiently implement the nursing content and improve the nursing effect. This paper studies the application of the PDCA nursing model in the nursing of children with Henoch-Schonlein purpura and statistically analyzes the disappearance of skin rash, joint pain relief, disappearance of urine protein, disappearance of gastrointestinal symptoms, etc. Finally, this paper combines the experiment to evaluate the intervention effect of this nursing model and provides reference for the follow-up care of children with Henoch-Schonlein purpura. From the results of experimental research, it can be known that PDCA nursing can improve the comfort of children with Henoch-Schonlein purpura, shorten the time for symptom disappearance, and speed up the recovery process.

## 1. Introduction

Henoch-Schonlein purpura (HSP) is a common paediatric diffuse small artery allergy condition that often affects the skin, digestive system, joints, kidneys, and other organs. While the majority of children with HSP have a favourable prognosis, the condition is prone to recur. In youngsters, repeated sickness might result in kidney damage. Additionally, the more recurrences, the more severe the impairment of kidney function. Around one-third of HSP patients develop Henoch-Schonlein purpura nephritis (HSPN), which results in renal injury [1].

The study's findings suggest that the prevalence and progression of HSP illness may be connected to children's poor lifestyles, which include an improper diet and excessive activity. As a result, we may enhance children's everyday lives to reduce the onset, development, and recurrence of HSP illness [2].

HSP is most prevalent in school-aged children between the ages of 3 and 14, and it affects more males than girls. The incidence of black children is lower than that of white and Asian youngsters. The sickness is clearly seasonal, and it is more prevalent in the spring, autumn, and winter. In recent years, the prevalence of HSP in children has increased year after year, owing to a variety of variables such as the environment and everyday interaction. Annual prevalence of HSP in children has been estimated to be as high as 20/100,000 [3], with severe cases being more prevalent. It was decided in 2006 that HSP should be classed as rheumatic illness. In 2012, during the Chapel Hill conference, the new vasculitis naming consensus formally changed the name of HSP to IgA vasculitis (IgAV). HPS manifests as diffuse abdominal distension associated with discomfort, rheumatoid arthritis or arthralgia, and/or kidney involvement, and biopsy reveals significant IgA deposition [4]. At the moment, the pathophysiology of HSP remains unknown. However, research suggests that it is associated with an aberrant immunological response, inflammation-induced damage, altered blood coagulation function, and hereditary variables. In recent times, it is considered that a more definitive pathophysiology for HSP is as follows: problems of humoral and cellular immune function, elevated IgA levels, and changes in the number of lymphocytes, lymphocyte subsets, and activities.

The article "Analysis of Nursing Effect of Children with Henoch-Schonlein Purpura Based on the PDCA Nursing Model" was retracted in 2022. Reason: concerns about the peer review.

Clinically, HSP is usually divided into five types: simple skin type, abdominal type, joint type, kidney type, and mixed type. More than half of the children have gastrointestinal reactions. The most common manifestation is abdominal pain and pain. Others may have vomiting and gastrointestinal bleeding, which may be due to vasculitis causing intestinal flora disorder and intestinal wall hemorrhage. About 2% of children appear acute gastrointestinal bleeding. 15% to 25% of children may be affected by joints, prone to arthralgia or arthritis. Severe kidney illnesses such as acute nephritis, nephrotic syndrome, and renal failure affect around 5% of the population. Although neurological symptoms like as headaches are uncommon in children with HSP, they sometimes occur. Children with aberrant emotions often exhibit high levels of excitement. HSP is a recurrent condition. Around 67.1 percent of children with HSP relapse after a year, according to relevant data. Repeated sickness may impair a child's renal function. The larger the number of recurrences, the more severe the impairment to kidney function. Judging from the current clinical symptoms, the children with recurrent episodes mainly appear in two forms: recurrence of rash and recurrence of nephritis. More and more studies have found that the prognosis of HSP mainly depends on the severity of kidney involvement, although diseases of organs other than the kidneys such as the brain and testes can sometimes lead to serious complications. HSP is not entirely a self-limiting disease. It has become one of the main causes of chronic kidney disease in children. The main manifestations are persistent proteinuria, hematuria, nephrotic syndrome, and even acute renal insufficiency and renal failure. Approximately 30% of children with HSP will affect the kidneys, and as many as 20% of children with HSPN will eventually cause kidney damage in children with chronic kidney disease. The prognosis of the kidneys in adults with chronic kidney disease is worse. The proportion of adults who progress to chronic renal insufficiency is higher than that of children.

The article "Analysis of Nursing Effect of Children with Henoch-Schonlein Purpura Based on the PDCA Nursing Model" was retracted in 2022. Reason: concerns about the peer review.

In order to improve the nursing effect of children with HSP, this paper combines the PDCA nursing model to analyze the effect of nursing intervention for children with HSP and evaluate the intervention effect of this nursing model with experiments, so as to provide references for subsequent nursing of children with HSP.

## 2. Related Work

Literature [5] found through meta-analysis that skin manifestations, such as persistent purpura and purpura rash, are significantly related to HSPN. Children with persistent purpura rash are 1 to 13 times more likely to develop HSPN than non-persistent ones, and children with recurrent rashes are 2.7 to 11 times more likely to develop kidney damage than non-recurrent rashes. There is no rigorous evidence for the duration. Some scholars claim that the duration of persistent rash is 1 month, and the number of repetitions of the rash mostly believes that 3 times or more than 3 times are related to HSPN. It may be that the continuous inflammation of small blood vessels expands a series of inflammatory reactions, induces immune-mediated reactions, and ultimately damages the kidney tissue. Some scholars have studied the risk factors of children with relapsed HSP and children with relapsed HSP and found that uncontrolled diet, respiratory infections, strenuous exercise, and other factors are risk factors for HSP recurrence [6].

Contemporary scientists think that food allergies mediated by IgE are associated with the start of HSP, which may affect the skin, respiratory system, and digestive tract, leading in skin itching, dyspnea, nausea, and vomiting. Recent research has shown that food intolerance, as mediated by IgG, plays a critical role in the development of HSP [7]. At the moment, the mechanism behind food intolerance is unclear. HSP and food intolerance testing revealed that foreign proteins such as eggs, milk, and beef are significant factors in the onset and recurrence of HSP, and children with relapsed HSP acquire sensitivity to other foods, suggesting recurring assaults. The body's harm is escalating [8]. Infection is also linked to the occurrence of HSP in youngsters. Upper respiratory tract infection is the most prevalent, followed by pneumococcal infection and urinary tract infection. The invasion of microorganisms into the body is linked to upper respiratory tract illness, as well as diminished body resistance and nutritional deficits. Poor eating habits and diet structure have been linked to frequent upper respiratory tract infections in local children and newborns, according to the literature [9]. Some patients have had substantial therapeutic outcomes by adding trace elements and multivitamins in the treatment of respiratory infections. Chinese medicine believes that food allergies are similar to “fengxie”, both of which are exogenous pathogens, and the characteristics of skin symptoms caused by invading the human body are similar. The rapid onset of food allergy is similar to the characteristics of “winds that are good and changing.” Some foods play a pivotal role in the body's allergies caused by “wind evil.” “Shrimp, flat, and scabies caused by wind,” and ingestion of products that move wind can induce “wind evil” to cause disease and cause the body to become abnormal. Reaction [10]. Modern Chinese medicine practitioners often add antiwind drugs such as Fangfeng to the treatment of HSP or other allergic diseases, which can treat the disease, because a variety of antiwind Chinese medicines have antiallergic effects and can inhibit the production of IgE [11]. This also demonstrates that the pathogenicity of “fengxie” is intimately linked to specific allergic disorders and that ingesting things that move the wind may readily trigger allergic responses.

The article "Analysis of Nursing Effect of Children with Henoch-Schonlein Purpura Based on the PDCA Nursing Model" was retracted in 2022. Reason: concerns about the peer review.

When modern scientists compare the physical characteristics of children with HSP to those of healthy children, they discover that children with HSP have the largest percentage of yin deficit, indicating that children with partial yin deficiency are more prone to HSP [12]. According to literature [13], the percentage of HSP children with a balanced TCM constitution was 36.94 percent, 33.78 percent had a partial yin deficit, and 53.57 percent had a partial yin deficiency, and the second was Qi insufficiency. The literature [14] analysis discovered that although the features, feeling, colour, density, and size of the rash varies substantially amongst children with various constitutions, it has no influence on the location of the rash and other concomitant symptoms. HSP rashes associated with yin deficient body are often bright red or purple in colour and are not associated with Itching, which is thicker and greater in diameter than other physique purpura.

## 3. Objects and Methods

Children with HSP who were treated in our hospital from November 2019 to June 2021 were chosen as study subjects, and they were separated into two groups based on nursing methods: a control group and an observation group. The two groups of youngsters had no statistically significant differences in general knowledge (*P* > 0.05), and they were comparable. All of the youngsters fit the diagnostic criteria for Henoch-Schonlein purpura in children. Furthermore, all children and their families were made aware of the research and freely completed an informed consent form. Exclusion criteria were as follows: children with obvious renal impairment and children with poor compliance.

The article "Analysis of Nursing Effect of Children with Henoch-Schonlein Purpura Based on the PDCA Nursing Model" was retracted in 2022. Reason: concerns about the peer review.

All children were given conventional treatments after the hospital, including glucocorticoids, immunosuppressants, anticoagulation therapy and antibiotics, and symptomatic and supportive treatments such as maintaining electrolyte balance and antipyretic analgesics were given to children when necessary. The control group was given routine care on the basis of routine treatment, such as inpatient environmental care, timely disinfection and ventilation of the ward, and prevention of cross-infection and nosocomial infection. In addition, the two groups of children also adopted the following nursing methods: (1) Psychological intervention nursing: when children are hospitalised, they develop negative emotions such as irritability and fear as a result of the unfamiliar hospital environment and the pain associated with the doctor's examination, operation, and treatment, which may result in crying and other situations. Mild cases will oppose examination and treatment, major cases will deny examination and treatment, and parents will experience worry and anxiety, which is not conducive to follow-up therapy. In response to this condition, nursing personnel must engage in psychological treatments with youngsters. Following the child's admission to the hospital, the nursing staff must actively and enthusiastically greet the children, patiently communicate and communicate with the children and their parents, earn the children's trust, and close the distance between the nursing staff and the children, all of which will alleviate the children's sense of strangeness and fear. Second, once the child is admitted to the hospital, it is necessary to arrange beds for the children as soon as possible, familiarise the children and their parents with the hospital environment, and explain disease inspection methods, treatment plans, and nursing measures to parents in an easy-to-understand language and with a cordial attitude. Furthermore, it is vital to minimize the children's strangeness and anxiety as soon as possible by playing games with them to help the children better adjust to the hospital environment and strengthen the children's and parents' collaboration. In addition, nursing staff should be as gentle as possible when performing physical examinations on children to avoid causing greater irritation to the children's body and encourage and praise the children during the operation. (2) Diet nursing intervention: the children's diet should be light and easy to digest, and ensure that there are sufficient fresh vegetables and fruits in the nursing diet. Because the child's body is in a state of hypersensitivity, children should avoid eating allergic foods. Nursing staff should carry out nutrition education and health education to parents, improve parents' awareness of nutrition knowledge, and assist parents in preparing reasonable meals for children. The order of food selection for children should be starchy foods first, followed by protein foods. If the child has obvious symptoms such as abdominal pain, vomiting, and blood in the stool, the child needs to fast for a period of time and be given intravenous nutritional support. If the child's abdominal pain, vomiting, and blood in the stool disappear after targeted treatment, the child can be given a liquid diet first. After that, depending on the child's condition, it is necessary to gradually transition to a normal diet. Simultaneously, the youngster needs vitamin C supplementation to minimise the fragility and permeability of the capillaries, which is favourable to the child's recuperation. Additionally, salt consumption should be restricted in children with impaired renal function. (3) Environmental nursing intervention: to reduce cross-infection and nosocomial infection in the hospital, personnel access and exit should be minimised, and nursing staff should clean, disinfect, and ventilate the ward on a regular basis. Simultaneously, it is vital to provide colourful cartoon toys and books in the ward to assure the children's happiness, as well as to play children's radio or music in the morning and midday to create a pleasant environment for the children. (4) Skin and oral care: the most common manifestation of allergic purpura in children is a rash on the skin. Children are immature, lack self-control, and are unaware of prevention. As a result, they often scratch the afflicted region, causing damage to the skin and increasing the risk of infection. As a result, nursing personnel should concentrate on caring for the child's skin, guiding parents to help if required, and applying the medication locally as directed by the doctor. To avoid infection when a rash or ulcer appears in the afflicted region, keep the skin dry and clean it on a regular basis. If the child's oral mucosa is affected, it is necessary to instruct the child to rinse the mouth with normal saline or wipe the affected area with a cotton ball before and after meals and before going to bed to keep the child's mouth clean. At the same time, it is important to remember to change children's bed linens and clothes on a regular basis to keep the body dry and limit the risk of infection. Theoretical management techniques are employed by nursing staff in the experimental group: each member of the experimental group must be taught in cyclic theory knowledge and work processes, and they must be freely applied in everyday nursing work. Moreover, members need to strictly demand themselves, be rigorous and realistic, develop good working habits, do every job in strict accordance with the step plan, and earnestly achieve the goals required by the PDCA cycle, and do self-inspection and mutual inspection. At the same time, the nursing department needs random inspections and the departments need regular self-examinations, and the composition of the experiment needs to form a good atmosphere for everyone to manage. The small cycle of each person in the experimental group merges with the entire large cycle of the experimental group as a whole, thereby promoting the large cycle of the entire experimental group to spiral upward in a spiral of steps, repeating itself again and again. The four stages are closely connected and inseparable. Planning, execution, and inspection are all interconnected in the real work process, and the inspection, summary, and adjustment processes all complement one another. The particular method is to provide work goals in order to identify existing issues, evaluate relevant causes, design appropriate plans, execute appropriate actions, monitor implementation impacts, and summarise experience and lessons learned or progress to the next cycle. The control group employs standard empirical management techniques, and each member closely adheres to nursing routines, enhances business learning, and requires random inspections by the nursing department.

(1) Stage P of planning (Plan). During routine inspections of the nursing department and departments, problems with the experimental group nurses' basic technical operations were carefully identified, pointed out to examinees on the spot, and corrected, and existing problems were sorted, summarised, and analysed and reported to the nursing department. The nursing department arranges the evaluation of fundamental nursing technical operations, and the invigilator promptly identifies and corrects the evaluated nurses' deficiencies, scores them on the spot, organises and analyses the issue records, and reports to the nursing department. The following are some of the most common reasons: (1) nurses have a poor understanding of basic operating standards and standards and have a poor concept of sterility; (2) the nurse has a poor concept of love and injury, the operation is blunt, the patient is not observed in time, and the problem cannot be dealt with in time; (3) during peak periods of work, individual nurses are not very responsible and often simplify the operation process of nursing technology; (4) before the operation, the nurses were underevaluated. It is necessary to formulate measures to address the problems in the assessment, analyze the reasons in time, summarize and summarize, and report to the nursing department. After that, the nursing department uniformly strengthened the training of the “Shandong Technical Operation Quality Evaluation Standards” for the nursing staff of the experimental group, so that everyone is proficient in the evaluation standards. At the same time, according to the situation of each member, the head nurse proposed targeted rectification measures for each person's different problems. In addition, each member of the experimental group must be proficient in operating standards, make continuous improvements in response to their own problems, and increase or decrease staff on duty according to the workload. (2) Implementation stage D (Do). The nursing department needs to strengthen the nursing technical operation training for the nursing staff of the experimental group, and ask the expert group for on-site guidance, and the nursing department and the expert group members will unify the standards and conduct unified operation demonstrations. It is necessary to carefully explain and demonstrate the handling and detailed requirements of the three key links before operation, during operation, and after operation. In the operation of basic nursing technology, the system of three checks and nine verifications and the principles of aseptic technique operation are emphasized from beginning to end. The nursing department sets up special personnel to supervise the technical operations, and the expert group members and the nursing department provide on-site guidance until each member of the experimental group is proficient. Under the unified organization of the nursing department, the nursing staff of the experimental group learned human science knowledge, such as laws and regulations, communication skills, and nurse etiquette, so that the overall quality of the experimental group was improved. Nursing staff actively evaluate patients before operation, attach importance to communication and communication with patients and their families, keep abreast of the ideological trends of patients and their families, and earnestly achieve empathy. During the operation, the nursing staff needs to observe the patient's reaction and needs in time and make appropriate treatments to the problems that arise. After the operation, the nursing staff needs to explain the precautions to the patient and family members in detail. (3) Check stage C (check). Every month, the system of the nursing department randomly draws all members of the experimental group and the control group and uses the on-site lottery method for assessment. Moreover, it is necessary to implement expert group invigilation and on-site scoring methods. Given the issues, on-site assistance is required, as well as a summary of prevalent concerns and a report to the nursing department. The issues that occur will be reviewed in the following cycle, and the nursing department will be in charge of overseeing them. Individual assistance is provided by the head nurse, who pushes correction of any personality issues that appear throughout the evaluation. Simultaneously, the head nurse must perform an indoor evaluation of the nurses in the overall experimental group in order to quickly resolve the issues reported by the nursing expert group during the assessment. During the evaluation process, nurses may also learn about other people's strengths and weaknesses, as well as grasp the assessment guidelines. After the assessment is over, it is necessary to immediately discuss the problems that occurred in the assessment, analyze the common and individual problems in the assessment, and propose corresponding specific rectifications. During the assessment process, it is necessary to emphasize the nurse's humanistic care for the patient, respect the patient and family members, always take the patient as the center, strengthen nurse-patient communication, and enable the patient and family members to truly have the right to decide and inform and achieve a win-win situation for improving nursing quality management and patient satisfaction. (4) Action stage A. The nursing department uniformly corrects the common problems found in the assessment, organizes training uniformly, and continuously improves and at the same time starts the next cycle. At the same time, it is necessary to select outstanding candidates to participate in various nursing skill competitions in the city and the whole hospital, and put the existing unresolved problems into the next cycle [15]

Circulation Management in Nurses' Hand Hygiene Research (1) Recognize Plan P (Plan) Contact transmission is a major mode of pathogen distribution in hospital infections, and the hands of medical workers constitute a significant mode of transmission in hospital infections. The hospital infection rate due by insufficient hand washing by medical workers is as high as 30%, and hand washing may drastically cut hospital infection rates by 50%, while also being less expensive. As a result, hand hygiene has evolved into the most direct, straightforward, economical, and successful method of preventing hospital infections. Recent studies, however, indicate that the efficiency of handwashing by medical personnel in my country is dubious. According to published accounts, 200 nurses were probed for improper handwashing. According to the study's findings, handwashing covers 32.5 percent of the processes and only 20.5 percent of the steps are qualified [16]. Reasons are analysed The following are the explanations behind the aforementioned issues: They have not received systematic training on hand washing knowledge, which results in nurses lacking hand washing knowledge; due to a lack of legal knowledge and hospital infection knowledge, nurses in outpatient infusion rooms have a relatively low level of awareness; the work of outpatient infusion centres is cumbersome; the workload is high, the time is limited, and there is little time to wash hands; no corresponding hand-washing or hand-drying facilities are provided. Make a list of measurements. The department organizes the experimental group nurses on a regular basis to reinforce the study of “Disinfection Technical Specifications,” “Nominal Infection Management Specifications,” and knowledge of laws and regulations, risk management knowledge, and other topics, as well as to improve hand-washing technology training and learn the “six-step hand-washing method” correctly and systematically. To enhance the monitoring and management of hand washing quality, a disinfection and isolation quality monitoring team was developed to be responsible for the hand quality monitoring and management of the experimental group nurses and hand washing quality testing, among other things. (2) In the implementation stage D (Do), under the unified organization of the nursing department, further change the quality control method, formulate and implement a “hand washing system”, strengthen hand washing awareness, post “hand washing behavior warnings” in actual work, and improve hand washing facilities and usage [17]. Things. Uniformly adjust the organization structure of disinfection and isolation quality management in the outpatient infusion center, and set up a “disinfection and isolation quality management leadership group” centered on the head nurse to be responsible for the quality monitoring and management of nurses' handwashing in the center. (3) Inspection stage C (check) handwashing effect monitoring includes Samples are taken immediately before operation and after washing hands, and the nursing department will conduct uniform monitoring and sampling of hand hygiene once a month [18]. The evaluation standard of hand washing technology refers to the “Disinfection Technical Specification”, the sampling method adopts the method specified in the “Disinfection Technical Specification”, and the judgment of eligibility is based on the requirements of the “Disinfection Technical Specification.” It is the criterion of judgment [19]. (4) Treatment stage A (action) standardizes hand hygiene, so that all nurses in the experimental group are proficient in the “six-step hand washing method”, and the head nurse supervises the implementation of hand washing every day. Discover new existing problems, formulate continuous quality improvement measures, and incorporate them into the next management cycle, to praise and reward nurses with high compliance with hand washing [20].

The article "Analysis of Nursing Effect of Children with Henoch-Schonlein Purpura Based on the PDCA Nursing Model" was retracted in 2022. Reason: concerns about the peer review.

## 4. Result

This paper statistically analyzes several aspects such as rash subsidence, joint pain relief, urine protein disappearance, and digestive tract symptom disappearance. The results obtained are shown in Tables 1–4 and Figures 1–4.

The pathogenesis of Henoch-Schonlein purpura is still unclear. It may be caused by infection, immune disorders and other factors that cause the body's immune complexes to deposit in the capillaries of the skin surface, which causes inflammatory reactions in the surrounding blood vessels. Moreover, it is often accompanied by complications such as joints, digestive tract, and kidney discomfort, and it mostly occurs in children. There is no specific medicine in clinical treatment, and the therapeutic effect is not ideal, and it is easy to recur, which seriously threatens the physical and mental health of children. In recent years, nursing has been widely used in clinical treatment, which can improve the treatment effect and promote the recovery of the body. Therefore, the application of nursing mode plays an important role in treatment. The results of this study showed that the comfort score of the observation group was lower than that of the control group, and the rash subsided, joint pain was relieved, urine protein disappeared, and the disappearance of digestive tract symptoms was shorter than the control group. It can be seen that PDCA nursing can improve the comfort of children with HSP and shorten the time for symptoms to disappear. The reason is that PDCA nursing is a more comprehensive nursing model, emphasizing on the care of patients' physiology, psychology, and human environment. It has systemic continuity and promotes patients to recover as soon as possible. Children with Henoch-Schonlein purpura for the first time and their family members, because of their obvious symptoms and lack of understanding of the disease, they are prone to fear in their hearts. In addition, repeated attacks can cause depression of the children and family members and affect their recovery. As a result, family members get health education so that they may have a clear grasp of the condition, relieve psychological stress, and gain treatment confidence, allowing them to actively participate in the treatment. Simultaneously, it is vital to develop a relaxing and pleasant treatment environment for children in order to limit external stimuli, prevent infection with other illnesses, and increase their comfort. The etiology of allergic purpura is more complicated and may be related to diet. Therefore, controlling diet and preventing accidental consumption of allergic foods play an important role in improving clinical symptoms and preventing disease recurrence, while also ensuring the body's nutritional balance. Patients with Henoch-Schonlein purpura have fragile skin, prone to itching, and poor self-control in children, so they often scratch their skin and cause infection. Therefore, skin care needs to be done to reduce bacterial infections and improve treatment efficiency. In addition, good symptom care can improve children's symptoms and relieve their pain, which is conducive to the prognosis. Timely review can observe the recovery of the condition and avoid recurrence. In summary, PDCA care can improve the comfort of children with HSP, shorten the time for symptom disappearance, and speed up the recovery process.

The article "Analysis of Nursing Effect of Children with Henoch-Schonlein Purpura Based on the PDCA Nursing Model" was retracted in 2022. Reason: concerns about the peer review.

## 5. Conclusion

Pediatric allergic purpura is an autoimmune disease. There are many causes of disease, including bacterial, viral, and parasitic infections; food such as milk, eggs, fish, and shrimp; antibiotics; antipyretic analgesics and other drugs; pollen allergies; and mosquito bites. These generate allergies in the child's delicate body, which produces self-antigens and antibodies, which subsequently form antigen-antibody complexes on the walls of tiny blood vessels throughout the body, causing vasculitis-related pathological changes. The poor compliance of pediatric nursing care has a stronger influence on nurse intervention in clinical nursing. Therefore, it is necessary to choose an appropriate nursing plan to intervene to improve the level and quality of care. Improper care is one of the main causes of allergic purpura in children. Improper care can easily lead to repeated illnesses and further affect the lives of children and their parents. The application of PDCA model in the diet and care of children with HSP has a significant effect. Therefore, it is possible to find an effective nursing path, improve the nursing plan, and improve the quality of nursing by analyzing the child's condition, eating habits, and nursing problems.

The article "Analysis of Nursing Effect of Children with Henoch-Schonlein Purpura Based on the PDCA Nursing Model" was retracted in 2022. Reason: concerns about the peer review.

## Figures and Tables

**Figure 1:** Histogram of rash subsidence time.

**Figure 2:** Histogram of joint pain relief time.

**Figure 3:** Histogram of urine protein disappearance time.

**Figure 4:** Histogram of the disappearance time of digestive tract symptoms.

**Table 1:** Test results of rash subsidence time.

Number	Test group	Control group	Number	Test group	Control group
1	2.81	2.78	21	2.48	3.29
2	5.05	4.05	22	3.26	3.02
3	1.14	3.06	23	3.31	4.78
4	4.74	3.74	24	1.38	5.95
5	5.63	5.78	25	3.18	4.10
6	4.33	5.05	26	1.83	4.47
7	2.58	5.23	27	2.57	3.81
8	4.94	5.43	28	1.47	6.05
9	3.79	5.45	29	5.57	4.04
10	4.68	3.37	30	4.78	3.63
11	1.02	3.28	31	2.72	5.33
12	4.67	5.75	32	2.23	3.83
13	5.72	5.24	33	3.83	3.06
14	2.77	5.54	34	4.14	6.15
15	3.05	6.38	35	2.54	4.20
16	3.10	2.82	36	2.14	4.64
17	3.28	5.90	37	1.83	6.71
18	2.92	5.24	38	0.67	4.97
19	3.36	2.42	39	3.46	5.62
20	4.27	2.90	40	3.33	6.55

**Table 2:** Test results of joint pain relief time.

Number	Test group	Control group	Number	Test group	Control group
1	4.33	4.48	21	4.15	5.33
2	3.48	3.07	22	4.69	5.35
3	2.63	4.80	23	4.56	4.75
4	3.25	5.05	24	3.53	4.49
5	4.06	5.29	25	2.90	5.12
6	4.12	4.20	26	3.79	4.59
7	2.64	3.93	27	2.73	3.03
8	2.77	4.19	28	4.76	5.11
9	3.02	5.19	29	4.65	5.08
10	3.67	3.78	30	4.82	5.48
11	4.02	3.61	31	3.58	4.40
12	2.99	3.79	32	3.16	4.86
13	3.11	3.05	33	2.49	4.54
14	4.83	3.85	34	3.56	4.06
15	4.70	4.25	35	2.63	5.68
16	4.33	3.27	36	2.54	3.03
17	3.77	4.39	37	4.17	3.82
18	2.64	4.46	38	3.37	3.94
19	2.77	3.99	39	4.09	5.32
20	4.30	3.71	40	4.72	3.24

**Table 3:** Test results of urine protein disappearance time.

Number	Test group	Control group	Number	Test group	Control group
1	13.03	14.73	21	11.27	12.72
2	13.11	12.28	22	12.44	15.55
3	12.23	14.46	23	11.72	11.13
4	13.07	14.03	24	12.94	13.00
5	13.11	12.28	25	12.55	13.49
6	13.17	11.23	26	11.61	11.47
7	12.94	11.87	27	12.02	13.85
8	11.31	14.50	28	11.45	11.54
9	12.33	12.50	29	13.25	14.24
10	11.70	16.09	30	12.13	13.01
11	13.08	11.15	31	11.29	11.70
12	13.18	14.77	32	12.81	11.01
13	11.24	13.29	33	11.22	12.58
14	12.01	15.48	34	11.88	14.10
15	11.82	13.93	35	12.07	13.60
16	11.61	13.00	36	13.46	12.83
17	11.13	15.56	37	13.19	11.05
18	13.43	14.08	38	12.54	11.92
19	11.83	12.28	39	11.42	14.25
20	13.39	12.45	40	12.69	12.79

**Table 4:** Test results of the disappearance time of digestive tract symptoms.

Number	Test group	Control group	Number	Test group	Control group
1	5.70	6.57	21	6.74	7.73
2	5.59	8.75	22	7.41	6.66
3	7.06	8.32	23	7.86	6.91
4	5.51	7.52	24	5.85	8.50
5	7.53	6.71	25	6.00	8.22
6	7.25	7.75	26	5.98	7.97
7	7.88	8.02	27	5.53	7.47
8	8.08	6.71	28	8.14	7.61
9	7.70	7.40	29	5.51	7.24
10	5.60	8.57	30	7.54	8.47
11	7.02	7.94	31	5.71	9.11
12	6.73	7.02	32	7.11	8.87
13	8.02	7.30	33	6.25	8.23
14	7.48	7.39	34	6.36	8.85
15	6.89	7.51	35	6.04	8.78
16	5.56	7.59	36	7.13	7.07
17	6.50	7.29	37	8.08	8.11
18	7.17	8.30	38	5.68	6.70
19	6.63	9.13	39	5.92	7.16
20	7.98	7.27	40	7.13	8.81

The article "Analysis of Nursing Effect of Children with Henoch-Schonlein Purpura Based on the PDCA Nursing Model" was retracted in 2022. Reason: concerns about the peer review.

## Data Availability

The data used to support the findings of this study are included within the article.
